The article "Succinylation Site Prediction Based on Protein Sequences Using the IFS-LightGBM (BO) Model" was published in 2020. Journal: Comput Math Methods Med.

# Succinylation Site Prediction Based on Protein Sequences Using the IFS-LightGBM (BO) Model

**DOI:** 10.1155/2020/8858489

**Published:** 2020-11-10

**Authors:** Lu Zhang, Min Liu, Xinyi Qin, Guangzhong Liu

**Affiliations:** College of Information Engineering, Shanghai Maritime University, 1550 Haigang Ave., Shanghai 201306, China

## Abstract

Succinylation is an important posttranslational modification of proteins, which plays a key role in protein conformation regulation and cellular function control. Many studies have shown that succinylation modification on protein lysine residue is closely related to the occurrence of many diseases. To understand the mechanism of succinylation profoundly, it is necessary to identify succinylation sites in proteins accurately. In this study, we develop a new model, IFS-LightGBM (BO), which utilizes the incremental feature selection (IFS) method, the LightGBM feature selection method, the Bayesian optimization algorithm, and the LightGBM classifier, to predict succinylation sites in proteins. Specifically, pseudo amino acid composition (PseAAC), position-specific scoring matrix (PSSM), disorder status, and Composition of *k*-spaced Amino Acid Pairs (CKSAAP) are firstly employed to extract feature information. Then, utilizing the combination of the LightGBM feature selection method and the incremental feature selection (IFS) method selects the optimal feature subset for the LightGBM classifier. Finally, to increase prediction accuracy and reduce the computation load, the Bayesian optimization algorithm is used to optimize the parameters of the LightGBM classifier. The results reveal that the IFS-LightGBM (BO)-based prediction model performs better when it is evaluated by some common metrics, such as accuracy, recall, precision, Matthews Correlation Coefficient (MCC), and *F*-measure.

## 1. Introduction

Posttranslational modification (PTM) is the chemical modification of the precursor protein after translation, such as the addition of a small molecule protein or the introduction of a functional group, so that the inactive precursor protein can obtain biological functions. There are many forms of posttranslational modifications of proteins, such as ubiquitination, glutarylation, sumoylation, palmitoylation, acetylation, and methylation. Succinylation is PTM that occurs on lysine. Lysine is an *α*-amino acid encoded by codons AAA and AAG and is easily modified [1]. Succinylation is a broadly conserved protein posttranslational modification that exists in prokaryotic and eukaryotic cells and can coordinate various biological processes [2–4]. Compared with the methylation and acetylation that occur on lysine, succinylation will cause more substantial changes in the chemical structure of lysine [5]. And in a variety of cell functions, including metabolism and epigenetic regulation, succinylated proteins are involved.

Some studies have shown that abnormalities and variations of succinylation associated with the pathogenesis of many diseases, including tumors [6–10], cardiac metabolic diseases [11, 12], liver metabolic diseases [13], and nervous system diseases [7, 14, 15]. Therefore, understanding succinylation and identifying the site of succinylation will help determine the pathogenesis of related diseases and develop targeted drugs [16].

Nowadays, many biological experimental methods have been developed to detect succinylated proteins or succinylation sites, such as the high-performance liquid chromatography assays, spectrophotometric assays, and radioactive chemical labeling [17, 18]. However, it is an arduous work on detecting protein succinylation through experiments, which inevitably waste lots of time and money. Machine learning, in contrast, has the advantage of performing a large number of experiments in a short time and has not been affected and restricted by external conditions, which are helpful on recognizing the succinylation sites. Zhao et al. [19] built a predictor called SucPred based on SVM using position amino acid weight composition, van der Waals volume normalized, grouped weight-based encoding, and autocorrelation functions. By using SVM, Xu et al. [20] developed iSuc-PseAAC that implemented a composition of pseudo amino acid (PseAAC) scheme. And then, Xu et al. [21] developed another predictor named SuccFind, which considered several amino acid-based composition encodings, including amino acid composition (AAC), *k*-spaced amino acid pairs (CKSAAP), and amino acid index (AAindex). Hasan et al. [1] proposed the approach SuccinSite predictor with the RF classifier by integrating multiple sequence features. Ning et al. [22] built a predictor called PSuccE based on SVM using amino acid composition (AAC), binary encoding (BE), physicochemical property (PCP), and grey pseudo amino acid composition (GPAAC).

Although many methods for predicting succinylation sites based on machine learning have been proposed, there is still much room for improvement based on machine learning. Firstly, the protein sequences' feature information is not clearly illuminated for predicting the effects of succinylation site interaction. Secondly, multi-information fusion produces high-dimensional feature vectors, which brings redundancy and noise information. There is an urgent need to use an efficient feature selection method to rank the importance of features and select the best feature subset from them. Finally, the development of experimental technology produced a large amount of succinylation data. How to make full use of experimental data to design effective prediction algorithms is very necessary.

In this study, we propose an IFS-LightGBM (BO) prediction framework based on machine learning to identify succinylation sites of lysines in protein sequences. Four sequence-based features are firstly used to represent the peptides: (1) pseudo amino acid composition (PseAAC), (2) position-specific scoring matrix (PSSM), (3) disorder status, and (4) Composition of *k*-spaced Amino Acid Pairs (CKSAAP). Secondly, the LightGBM method is used to prioritize the 2501-D feature vector, which obtains from these four sequence-based features. Thirdly, we combine the incremental feature selection (IFS) method and the machine learning methods to perform effective feature fusion and then determine the optimal feature subset, which can eliminate the noise and redundancy information in the original feature vector. Finally, the Bayesian optimization (BO) algorithm is used to optimize the parameters of the LightGBM classifier. This work provides not only a better understanding of the sequence characteristics of protein succinylation modification but also an effective algorithm for directly predicting the succinylation sites in proteins.

## 2. Materials and Methods

### 2.1. Dataset

In this work, the training data were collected from dbPTM [23, 24] (http://dbptm.mbc.nctu.edu.tw/index.php), which integrated published literatures, public resources, and a total of eleven biological databases related to PTMs. We obtained 2599 protein sequences including 5049 experimentally verified lysine succinylation sites and 5526 nonsuccinylation sites remained from dbPTM. The data in the dataset used a window size of 2*r* + 1 to extract the corresponding peptide fragment with lysine (K): “1” was a lysine (K) which was extracted as the central site of a polypeptide segment; “*r*” was equal to 10, which meant that 10 AA (amino acid) residues were selected from the upstream and downstream of lysine; and finally, a polypeptide segment with a length of 21 was obtained. Among them, the positive sample took the succinylated residue as the central site.

### 2.2. Description and Representation of Samples

Encode each polypeptide segment as a numeric vector and input it as a feature into the model. This is the most critical step in building an effective predictive model. Therefore, it is necessary to use high-quality sequence encoding methods to generate features that can effectively predict succinylation sites. In this study, we use four types of amino acid feature encoding methods including CKSAAP, disorder, pseudo amino acid composition, and PSSM.

#### 2.2.1. CKSAAP Encoding

The CKSAAP is one of the most classic encoding methods which has been widely used by people in bioinformatics tasks [1, 25–31]. In this study, we use polypeptide segments of length 21. Take AxA as an example, whose space number *k* is equal to 1. For the polypeptide segment which is composed mainly of 20 basic amino acids (i.e., A, R, D, C, ..., W, Y, V), when *k* = 0, the residue pairs that we need to extract are AA, AR, AD,..., VV, namely, there have a total of (20 × 20) = 400 amino acid pairs.

The following formula is used to calculate the feature vector:

(1) $$\begin{array}{c} {\left(\frac{N_{A,A}}{N_{\text{total}}},\frac{N_{A,R}}{N_{\text{total}}},\frac{N_{A,D}}{N_{\text{total}}},\cdots ,\frac{N_{V,V}}{N_{\text{total}}}\right)}_{400}, \end{array}$$

where *N*_*i*,*j*_ represents the number of amino acid pairs *i*, *j* with a distance of *k*, *N*_total_ is the total number of *k*-spaced residue pairs in the fragment. In this study, the optimal *k*_max_ is set as 4 (i.e., *k* = 0, 1, 2, 3, 4); then, the *N*_total_ will be 20, 19, 18, 17, and 16, which is obtained by calculating *N*_total_ = *L* − *k* − 1. Thus, a polypeptide segment with a length of 21 is transformed into a 2000-dimensional (400 × 5) AA composition feature vector.

#### 2.2.2. Disorder

One of the important indicators to measure the degree of protein structure is its inherent disorder. A large number of research results show that the inherent disorder of proteins plays a very important role in the prediction of protein structure and function [32–34]. In order to characterize this property, we use the VSL2B [35] program to predict the disorder score value. By running the tool, two types of results will be obtained, namely, qualitative and quantitative. The quantitative result is a value in the range [0, 1]. It is generally believed that 0.5 is the boundary value for distinguishing order and disorder. If the scoring result exceeds 0.5, it is considered disorder, otherwise order. For a polypeptide segment with a length of 21, the disorder features with 21-dimensional will eventually be obtained.

#### 2.2.3. Pseudo Amino Acid Composition (PseAAC)

In order to avoid complete loss of sequence-order information, the PseAAC [36] was proposed by Chou. PseAAC is an extended form of AAC, and it can identify salient hidden information [37–39]. In this work, Type-1 PseAAC is used as the dominating sequence representations. Let *A* be a polypeptide segment with the length of *L*, and *R*_*i*_(*i* = 1, 2, ⋯, *L*) is the *i*th residue of *A*:

(2) $$\begin{array}{c} A=R_{1},R_{2}\cdots R_{L}. \end{array}$$

The Type-1 PseAAC is a function of *A*, which produces a (20 + *λ*)-D vector. The mathematical formulation of Type-1 PseAAC is

(3) $$\begin{array}{c} P\left(A\right)={\left[p_{1},p_{2},p_{3}\cdots p_{20},p_{21},p_{22},p_{23}\cdots p_{20+\lambda }\right]}^{T}, \end{array}$$

where the first 20 features that can be obtained based on the composition of a given polypeptide segment, hydrophobicity, side-chain mass, and hydrophilicity of AAs are used to calculate the remaining *λ* features [38]. The *p*_*n*_ of *P* can be computed by Equations (4) and (5):

(4) $$\begin{array}{c} p_{n}=\left\{\begin{array}{c} \frac{f_{n}}{\sum_{i=1}^{20}f_{i}+w\sum_{j=1}^{\lambda }b_{j}}\left(1\leq n\leq 20\right),\\ \frac{{wb}_{n-20}}{\sum_{i=1}^{20}f_{i}+w\sum_{j=1}^{\lambda }b_{j}}\left(20<n\leq \lambda +20\right), \end{array}\right. \end{array}$$

(5) $$\begin{array}{c} b_{\lambda }=\frac{\sum_{i=1}^{L-\lambda }\left(1/3\right)\left[{\left(H_{1}\left(R_{i}\right)-H_{1}\left(R_{i+\lambda }\right)\right)}^{2}+{\left(H_{2}\left(R_{i}\right)-H_{2}\left(R_{i+\lambda }\right)\right)}^{2}+{\left(M\left(R_{i}\right)-M\left(R_{i+\lambda }\right)\right)}^{2}\right]}{L-\lambda }, \end{array}$$

where *f*_*i*_ reflects the occurrence frequency of the 20 standard amino acids, *b*_*j*_ is the *j*th tier sequence correlation factor, *ω* is the weight balance parameter for the sequence order effect, and *λ* is the lag parameter. *H*_1_(*R*_*i*_) and *H*_2_(*R*_*i*_) are normalized values of hydrophilicity and hydrophobicity, respectively. The normalized values of the side-chain mass of *R*_*i*_ are *M*(*R*_*i*_). Therefore, when *λ* = 20 and *w* = 0.05, each polypeptide segment is transformed into 40 dimensions AA composition feature vector.

#### 2.2.4. PSSM (Position-Specific Scoring Matrix)

Use PSI-BLAST [40] software to search against the SWISS-PROT database to obtain protein evolution information, where the BLAST local protein database is an authoritative protein database which is established by the University of Geneva and the European Bioinformatics Institute (EBI) [41]. By running the PSI-BLAST tool, two *L* × 20(*L* = 21) matrices can be obtained. The first one is the position-specific scoring matrix (PSSM), which is used to represent the conversation scores of 20 standard AAs occurring at specific sequence positions during evolution. The second one is the position-specific frequency matrix (PSFM), which contains the frequency of occurrence for a given amino acid at a specific sequence position. For the PSSM, we expand it into a 440-dimensional vector (420 + 20) in the following way. Firstly:

(6) $$\begin{array}{c} F_{\text{PSSM}}=\left[\left(S_{1_{A}},S_{1_{R}},\cdots ,S_{1_{V}}\right),\cdots ,\left(S_{L_{A}},S_{L_{R}},\cdots ,S_{L_{V}}\right)\right]. \end{array}$$

In addition, *F*_PSSM−mean_ features can be extracted from the PSSM:

(7) $$\begin{array}{c} F_{\text{PSSM}-\text{mean}}={\left[\frac{\sum_{i=1}^{L}S_{i_{A}}}{L}\frac{\sum_{i=1}^{L}S_{i_{R}}}{L}\cdots \frac{\sum_{i=1}^{L}S_{i_{V}}}{L}\right]}^{T}, \end{array}$$

where *L* is the length of each polypeptide segment, *S*_*ij*_(*i* = 1, ⋯, *L*; *j* = 1, ⋯, 20) is the values in the matrix. The features of PSSM are achieved by the integration of *F*_PSSM−mean_ and *F*_PSSM_.

We combine four characterizations to obtain a total of a 2501-D feature vector from each polypeptide segment. The distribution of the 2501 features is listed in Table 1. Then, several kinds of feature selection method will be used to rank the 2501-dimensional features according to their importance.

### 2.3. Feature Selection Method

Before models are developed, because the dataset may have features that are unrelated to target value or noise interfered, it is necessary to select the optimal feature subset through feature selection, so as to reduce the dimension of feature space to further decrease the risk of overfitting. At the same time, the generalization performance and the prediction ability of the models can be further improved when irrelevant features are removed ahead of training. In this article, the LightGBM feature selection method is used to select independent variables that are used to form the optimal feature subset.

LightGBM is an effective GBDT implementation algorithm, which is designed by Microsoft Research Asia [42]. For the LightGBM algorithm, two kinds of the importance type are contained: one is the “split” and the other is “gain.” “Split” reflects the number of times the feature is used in a model. When building the boosted trees, the important features are used more frequently, and the rest are used to improve on the residuals. In this study, the importance type is “gain.” Different from the “split,” the “gain” measures the actual decrease in node impurity. The feature rankings of gain-based importance can be obtained after LightGBM fitting [43].

### 2.4. Incremental Feature Selection Method

The combination of the IFS method and feature selection method is helpful to select the optimal feature subset. First, the feature selection method is used to construct the feature list. Specifically, different feature selection methods will firstly generate the importance scores of all features in light of the calculation criteria, then arrange the features in descending order according to the importance scores, and finally construct a corresponding feature list based on the importance scores, where the feature list is denoted as *F* = [*f*_1_, *f*_2_, ⋯, *f*_*L*_](1 ≤ *L* ≤ 2501). Next, incremental feature selection (IFS) [44] makes a series of feature subsets. IFS is a process of building an increasing number of feature subsets by gradually adding features. In this study, the incremental step length of the IFS method is set to 1, thereby constructing a series of feature subsets which can be denoted as FS_*m*_^1^, FS_*m*_^2^, ⋯, FS_*m*_^*L*^, in which the feature subset of FS_*m*_^1^ is constructed using the features ranked first in the feature list, and FS_*m*_^2^ has the top 1 and top 2 features, namely, FS_*m*_^*i*^ = [*f*_1_, *f*_2_, ⋯*f*_*i*_](1 ≤ *i* ≤ *L*). Then, the generated feature subsets are sequentially input into the classifier, which use the 10-fold cross-validation method to evaluate. Finally, when the fitness function of the predictor uses a certain feature subset to reach its maximum value, its corresponding feature subset is the best feature subset.

### 2.5. LightGBM

LightGBM is an algorithm that has been successfully applied in the field of classification, ranking, and many other ML tasks [43, 45–48]. It is an ensemble model based on a decision tree algorithm. In order to reduce memory usage and increase the training speed, the Histogram Algorithm is used in LightGBM, which tries to discretize every feature (successive floating-point eigenvalues) in the dataset into *k* small bins. After that, these bins are used to construct the histogram with width *k*. Once all the samples are traversed, the histogram will accumulate the required statistics that are gradients and number of samples' in each bin. After accumulating these statistics, the optimal segmentation point can be found based on the maximum gain provided when *k* bins are divided into two parts.

Besides Histogram Algorithm, LightGBM proposes gradient-based one-side sampling (GOSS), exclusive feature bunding (EFB), and leaf-wise growth methods to further improve computational efficiency without hurting the accuracy. When finding the best split in GOSS, the absolute value of samples' gradients is firstly used to sort the data instances. Then, preserve data instances with higher gradients, and randomly sample instances with low gradients. Finally, GOSS calculates the variance gain ${\tilde{V}}_{j}\left(d\right)$ of feature *j* to give the best split node.

(8) $$\begin{array}{c} {\tilde{V}}_{j}\left(d\right)=\frac{1}{n}\left(\frac{{\left(\sum_{x_{i\in A_{r}}}g_{i}+\left(\left(1-a\right)/b\right)\sum_{x_{i\in B_{l}}}g_{i}\right)}^{2}}{n_{l}^{j}\left(d\right)}+\frac{{\left(\sum_{x_{i\in A_{r}}}g_{i}+\left(\left(1-a\right)/b\right)\sum_{x_{i\in B_{l}}}g_{i}\right)}^{2}}{n_{l}^{j}\left(d\right)}\right),\\ \left\{\begin{array}{c} A_{l}=\left\{x_{i}\in A:x_{ij}\leq d\right\},A_{r}=\left\{x_{i}\in A:x_{ij}>d\right\},\\ B_{l}=\left\{x_{i}\in A:x_{ij}\leq d\right\},B_{r}=\left\{x_{i}\in A:x_{ij}>d\right\},\\ n_{l}^{j}\left(d\right)=\sum I\left(x_{i}\in \left(A_{l}\cup B_{l}\right)\right),\\ n_{r}^{j}\left(d\right)=\sum I\left(x_{i}\in \left(A_{r}\cup B_{r}\right)\right), \end{array}\right. \end{array}$$

where *A* is the instance set with high gradients and *B* is the instance set with low gradients. *g*_*i*_ is the gradients of each sample, *a* is the sampling ratio of large gradient data, *b* is the sampling ratio of small gradient data, and *d* is the number of iterations.

Furthermore, EFB can speed up the training process of GBDT via bundling exclusive features into a single “big” feature. Compared with the level-wise growth strategy, the leaf-wise growth strategy will choose the leaf with max delta loss to grow, which can reduce more errors and obtain better accuracy under the same splitting times.

### 2.6. Model Construction and Performance Evaluation

For convenience, the succinylation site prediction method proposed in this study is called IFS-LightGBM (BO). The use of flowcharts can more intuitively show the internal mechanism of model construction. Therefore, we draw Figure 1 to show the overall framework of IFS-LightGBM (BO). The framework is implemented using PyCharm 2020 and Python 3.6. The experiment is conducted on a computer with 2.30 GHz, 32.0 GB RAM, and Windows operating system.

The specific steps of IFS-LightGBM (BO) for the succinylation site prediction are described as follows:

1. *Dataset*. The dataset is used to predict succinylation sites, and it is divided into two categories: positive samples containing succinylation sites and negative samples without succinylation sites; the numbers are 5049 and 5526, respectively
2. *Feature Extraction and Feature Selection*. In this study, four feature extraction methods are used: PseAAC, disorder, PSSM, and CKSAAP, which transform the protein sequence signal into a numerical signal. For PSSM, two kinds of encoding methods are used, namely, averaged by column and expanded by row. Then, these four feature extraction methods are fused to predict the succinylation site. As what follows, the LightGBM method is used to prioritize the features and generate the feature list
3. *IFS-LightGBM (BO) Model Construction*. The IFS method builds a series of feature subsets based on the feature list, and then, the generated feature subsets are input into the LightGBM classifier in turn. The 10-fold cross-validation is used to evaluate the predictive ability of the classifier. When the performance of the classifier reaches the best, the corresponding feature subset is the optimal feature subset. The selected best feature subset is used as the input features of the model, and then, the BO algorithm is used to optimize the hyperparameters of IFS-LightGBM (BO). Five measurement metrics including ACC and *F*-measure are used to evaluate model performance

Protein PTM site prediction is essentially a binary classification problem, which can be measured using the notation in Table 2.

TP and FP represent the numbers of true positive and false positive, and the numbers of true negative and false negative are represented by TN and FN, respectively. To evaluate the prediction performance of our proposed method, five measures including accuracy (ACC), recall, precision, Matthews Correlation Coefficient (MCC), and *F*-measure are used [49]. These metrics are calculated as follows:

(9) $$\begin{array}{c} \text{Accuracy}=\frac{\text{TP}+\text{TN}}{\text{TP}+\text{FP}+\text{TN}+\text{FN}},\\ \text{Recall}\left(\text{sensitivity}\right)=\frac{\text{TP}}{\text{TP}+\text{FN}},\\ \text{Precision}=\frac{\text{TP}}{\text{TP}+\text{FP}},\\ \text{MCC}=\frac{\text{TP}\times \text{TN}-\text{FP}\times \text{FN}}{\sqrt{\left(\text{TP}+\text{FP}\right)\left(\text{TP}+\text{FN}\right)\left(\text{TN}+\text{FP}\right)\left(\text{TN}+\text{FN}\right)}},\\ F‐\text{measure}=\frac{2\times \text{Precision}\times \text{Recall}}{\text{Precision}+\text{Recall}}. \end{array}$$

ACC describes the proportion of samples that is correctly predicted, and its value ranges from 0 to 1, where 1 indicates the best prediction. Recall is the ability to identify positive cases, and precision denotes the class agreement of the data labels with the positive labels given by the classifier. MCC is a correlation coefficient describing the relationship between actual classification and predicted classification. *F*-measure can combine recall and precision into a single class-specific accuracy, which is selected as the key measurement in this study.

## 3. Results and Discussion

### 3.1. Integrated Optimal Feature Extraction

CKSAAP characterizes the short sequence motif information of polypeptide segments, PSSM reflects evolutionary information, disorder features reflect natively disordered residues recognized by VSL2B [35], and PseAAC reflects the physicochemical information of polypeptide segments. Therefore, it is possible that the integration of such four kinds of encodings will characterize the sequence and structural features of polypeptide segments better. But at the same time, the dataset after feature fusion may have features that are unrelated to the target value, so the LightGBM ranking algorithm will be used to sort the fused features and generate a feature list, and then, the IFS method will be used to select the optimal feature subset. This section uses 10-fold cross-validation to evaluate the performance of the model. The corresponding results are shown in Table 3. “All (IFS)” represents the fusion of the four feature extraction methods and the dimensionality reduction through the IFS and LightGBM feature selection method. “All” represents the fusion of the four feature extraction methods without dimensionality reduction.

It can be seen that when using the PseAAC, disorder, CKSAAP, PSSM, and “All” feature extraction methods, the *F*-measure scores are 69.37%, 56.79%, 68.29%, 67.56%, and 71.03%, respectively. The prediction *F*-measure of “All (IFS)” is 72.32%, which is 1.29% higher than that of “All” and 15.53% higher than that of disorder. We can clearly see that when the four feature extraction methods are fused, as well as the IFS and LightGBM are used to select the optimal feature subset, the prediction *F*-measure is significantly improved. Moreover, we can see that the prediction accuracy of “All (IFS)” is 2.99%, 16.51%, 3.96%, 3.75%, and 1.07% higher than those of PseAAC, disorder, CKSAAP, PSSM, and “All.” In summary, fusing the four feature extraction methods and using IFS and LightGBM to select the optimal feature subset can improve the prediction performance of protein succinylation sites. Hence, we combine the four feature extraction methods of PseAAC, disorder, CKSAAP, and PSSM to characterize information of each polypeptide segment.

### 3.2. Results of the IFS and Feature Selection Methods

Using multiple feature extraction methods can better characterize polypeptide segments, but at the same time, it will increase the risk of feature redundancy. In order to select the optimal features, the combination of the IFS method and different feature selection methods will be introduced. Meanwhile, in order to clearly reflect the superiority of the LightGBM feature selection method, we also use ReliefF [50], LinearSVR [51], XGBoost [52], and ANOVA [53] to find the optimal feature subset.

It can be seen from Table 4 that for the dataset, different feature selection methods have a great impact on the accuracy of succinylation site prediction. Among them, the LightGBM feature selection method enables the classifier to obtain the best prediction performance. When the top 351 features are selected as the feature subset, the ACC, recall, precision, MCC, and *F*-measure are 73.60%, 72.23%, 72.40%, 47.08%, and 72.32%, respectively. The *F*-measure of LightGBM is 0.51%, 0.73%, 0.04%, and 0.56% higher than that of ReliefF, LinearSVR, XGBoost, and ANOVA, respectively. The ACC is 0.41%, 0.56%, 0.09%, and 0.44% higher than that of ReliefF, LinearSVR, XGBoost, and ANOVA, respectively. The number of optimal features of LightGBM is 1963, 1756, 212, and 852 less than that of ReliefF, LinearSVR, XGBoost, and ANOVA, respectively. Furthermore, we also try the dimensionality reduction methods of the principal component analysis (PCA) [54] and *t*-Distributed Stochastic Neighbor Embedding (t-SNE) [55] without using the IFS method. As we can see from Table 4, when PCA is used to select the best feature subset, the *F*-measure value of the model is 0.6746, which is 4.86% less than LightGBM and 4.13% less than LinearSVR. Meanwhile, when*t*-SNE is used to select the best feature subset, the *F*-measure value of the model is 0.5218, which is 20.14% less than LightGBM and 19.41% less than LinearSVR. The experimental results indicate that although they consume less time, their predictive performances are worse than using other feature selection methods which combined with IFS, when processing the data in this study. Thus, we choose the way in combining IFS with different feature selection methods to select the optimal feature subset.

To further analyze, we draw the IFS curve plots of the predicted values for each feature selection method (i.e., LightGBM, ReliefF, LinearSVR, XGBoost, and ANOVA) as shown in Figure 2. It can be seen from Figure 2(b) that the LightGBM achieves the optimal *F*-measure result through a subset with 351 features, while the ReliefF, LinearSVR, XGBoost, and ANOVA achieve the optimal *F*-measure value when using the subset of the top 2314, 2107, 563, and 1203 features in their own feature list, respectively. Meanwhile, the LightGBM achieves the optimal ACC result using the subset of the top 351 features, while the ReliefF, LinearSVR, XGBoost, and ANOVA achieve the optimal ACC value when using the subset of the top 1465, 2130, 421, and 1203 features in their own feature list, respectively. In this section, the feature lists are different because these feature lists are constructed through different feature selection methods, but the feature subsets generated based on the feature lists will be input to the same classifier. The number of features used in the optimal feature subset determined by the LightGBM method is the least, while its corresponding ACC and *F*-measure scores are the highest. Conversely, the best feature subset of the LinearSVR contains the largest number of features, and its prediction accuracy and *F*-measure are smaller. Given the above, the prediction effect of the LightGBM feature selection method is better than ReliefF, LinearSVR, XGBoost, and ANOVA. Thus, we use the LightGBM feature selection method to select the best feature subset.

### 3.3. Selection of Classification Algorithms

The choice of classifier plays a crucial role in constructing an effective prediction model of succinylation sites. According to the discussion in Section 3.1, the 2501-dimensional feature vector will be obtained by fusing four feature extraction methods including PseAAC, disorder, CKSAAP, and PSSM. According to the analysis in Section 3.2, LightGBM will be used as the feature selection method and combined with the IFS method to construct the optimal feature subset. For the sake of reflecting the superiority of the LightGBM classifier in predicting succinylation sites clearly, Random Forest (RF) [56], ExtraTree (ET) [57], Gradient Boosting Decision Tree (GBDT) [58], *k*-nearest neighbor (kNN) [59], XGBoost, and Naïve Bayes (NB) [60] algorithms will be introduced and compared with it. The number of neighbors in kNN is 5, the number of base decision tree in RF is 100, the number of iterations of LightBGM, XGBoost, and GBDT is 100. It can be seen from Table 5 that when the LightGBM classifier uses a subset of the top 351 features in the LightGBM feature list, the *F*-measure value can achieve the best classification performance, which is 0.7% higher than GBDT and 13.64% higher than ET. Meanwhile, the ACC value of the LightGBM classifier is 0.7360, which is 1.78%, 13.5%, 0.93%, 7.64%, 0.89%, and 4.82% higher than that of RF, ET, GBDT, kNN, XGBoost, and NB, respectively.

Moreover, Figure 3 depicts the IFS curves of the ACC value and *F*-measure value of each classifier. It can be seen from the curve in the figure that when a subset of the top 351 features in the LightGBM feature list is used by the LightGBM classifier, both the *F*-measure and ACC achieve the optimal classification performance. For RF, ET, GBDT, KNN, XGBoost, and NB algorithms, the highest *F*-measure values are obtained when they use the top 37, 33, 94, 32, 427, and 805 features in the LightGBM feature list, respectively. And when separately using the top 41, 9, 131, 16, 427, and 44 features in the LightGBM feature list, they can obtain the highest ACC.

To prove that the LightGBM classifier is better than the other six machine learning algorithms, we conduct 100 times 10-fold cross-validation on different classifiers by setting different random seed numbers for the cross-validation method, in which the optimal subsets constructed by IFS are acted as the trainset for training different classifiers. To further measure the performances of the seven machine learning methods, we calculate the mean of maximum ACC (Max_ACC mean), the mean of maximum *F*-measure (Max_*F*-measure mean), the standard deviation of the maximum ACC (Max_ACC std), and the standard deviation of the maximum *F*-measure (Max_*F*-measure std) of each classifier. The results are listed in Tables 6 and 7, respectively. As shown in Tables 6 and 7, the prediction performance of the LightGBM classifier is better than the other six machine learning methods because its “Max_*F*-measure mean” and “Max_ACC mean” are higher than the RF, ET, GBDT, kNN, XGBoost, and NB algorithms. The “Max_*F*-measure std” and “Max_ACC std” of NB are smaller than other algorithms, which show that it has a relatively stable prediction performance. It can be seen from Figure 4 that the results of *F*-measure basically fit the normal distribution, and the continuities of the evaluation metric distributions of the RF, GBDT, kNN, XGBoost, and NB are better than the LightGBM. And the maximum *F*-measure of the 100 experiments of the LightGBM method is concentrated between 0.712 and 0.718. In conclusion, the LightGBM model has a better predictive performance than the other six models. So, we use LightGBM as the classifier. Figure 4 describes the histogram of the results of the 100 experiments.

### 3.4. Parameter Tuning and Performance Analysis

In order to further improve the performance of the LightGBM model, the Bayesian optimization (BO) algorithm is used to optimize the model parameters. Bayesian optimization is an extremely powerful method, which uses a surrogate function to estimate the noisy, expensive black-box functions. The core idea of the Bayesian hyperparameter optimization algorithm is to establish a probabilistic model that defines a distribution over objective functions from the input space to the objective of interest [61]. BO uses prior knowledge to approach the relatively cheap posterior distribution and then infers where to explore the next optimum hyperparameter combination according to the distribution. In this study, the Gaussian process (GP) approach is selected as a surrogate model and Expected Improvement (EI) is selected as an acquisition function.

For the surrogate model hyperparameters Θ, let *D* = {(*x*_*n*_, *y*_*n*_)_*n*=1_^*N*^} be the observations of input-target pairs, *σ*^2^(*x*; *D*, Θ) be the predictive variance function, the predictive mean value is *μ*(*x*; *D*, Θ), and define

(10) $$\begin{array}{c} a_{\text{PI}}\left(x;D,\Theta \right)=\Phi \left(\gamma \left(x\right)\right),\\ \gamma \left(x\right)=\frac{f\left(x_{\text{best}}\right)-\mu \left(x;D,\Theta \right)}{\sigma \left(x;D,\Theta \right)},\\ a_{\text{EI}}\left(x;D,\Theta \right)=\sigma \left(x;D,\Theta \right)\left[\gamma \left(x\right)\Phi \left(\gamma \left(x\right)\right)+\phi \left(\gamma \left(x\right)\right)\right], \end{array}$$

where *f*(*x*_best_) is the lowest observed value, Φ and *ϕ* are the standard cumulative and normal density, respectively [62].

The Bayesian optimization (BO) algorithm is used to optimize some critical hyperparameters in the LightGBM classifier as shown in Table 8. The *F*-measure between training values and predictive values of 10-fold cross-validation is defined as the fitness function evaluation of hyperparameter optimization of the LightGBM classifier. In order to distinguish from the LightGBM without hyperparameter optimized, the classifier which is optimized by the BO algorithm is called IFS-LightGBM (BO).

For the IFS-LightGBM (BO) model which uses the optimal feature subset with the 351 features, the parameters *learning_rate*, *max_depth*, *max_bin*, *reg_alpha*, *boosting_type*, *num_leaves*, and *n_estimators* need to be optimized by using the BO algorithm. The IFS-LightGBM (BO) model with the highest *F*-measure can be implemented when *learning_rate* is 0.0274, *max_depth* is 20, *max_bin* is 10, *reg_alpha* is 0.9647, *boosting_type* is goss, *num_leaves* is 11, and *n_estimators* is 600, which gave *F*-measure of 0.7255. For the sake of reflecting the superiority of the BO algorithm in tuning parameters clearly, we also employ a grid search (GS) method to optimize parameters of the LightGBM classifier, and the optimization process of the hyperparameters is shown in Table 9.  Table 10 lists other measurement results of IFS-LightGBM (BO), LightGBM, and IFS-LightGBM (GS). In Tables 10 and 11, “LightGBM (GS)” represents the model with the GS method; “LightGBM” represents the model without hyperparameter optimization.

To confirm that the performance of the LightGBM classifier has been further improved by the BO algorithm, we conduct 100 times 10-fold cross-validation on the IFS-LightGBM (BO) model. Meanwhile, the LightGBM classifier and LightGBM (GS) model are also evaluated by 10-fold cross-validation 100 times.  Table 11 shows the average and standard deviation of the maximum *F*-measure of three models for 100 random tests, which are IFS-LightGBM (BO), LightGBM, and LightGBM (GS). As can be seen from Table 11, the “Max_*F*-measure mean” of the IFS-LightGBM (BO) model is higher than the LightGBM (GS) model and LightGBM classifier. Meanwhile, compared with the grid search method, the Bayesian optimization algorithm has less time consumption in searching the optimal parameters for the LightGBM classifier. Therefore, the Bayesian optimization algorithm is used to optimize parameters of LightGBM to construct the optimal model.

Next, we will further analyze the model output results. On the basis of the output from Section 3.2, we find that when we use the subset of the top 351 features in the LightGBM feature list, the values of *F*-measure and ACC reach the highest point. It can be seen from Figure 5(a) that among the top 100 features in the feature list, the numbers of PseAAC, disorder, CKSAAP, and PSSM are 38, 16, 9, and 37, respectively. The evolution information (i.e., PSSM) and the physicochemical information (i.e., PseAAC) account for 38% and 37% of the total. Among the top 101-200 features in the feature list, the numbers of PseAAC, disorder, CKSAAP, and PSSM are 2, 5, 29, and 64, respectively. At the same time, among the top 201-351 features in the feature list, the numbers of CKSAAP and PSSM are 46 and 105, respectively.

## 4. Conclusions

The study of succinylation and its sites plays an important role in determining the pathogenesis of related diseases and the development of targeted drugs. In this study, we propose a model IFS-LightGBM (BO) based on machine learning for the prediction of succinylation sites. For the dataset, the PseAAC, disorder, PSSM, and CKSAAP four feature extraction methods are used to extract the sequence information and physicochemical information of polypeptide segments. At the same time, the IFS method and different feature selection methods are introduced and combined with the LightGBM classifier to eliminate redundant and noise information to determine the best feature subset. Through comparison, we find that compared with ReliefF, LinearSVR, XGBoost, and ANOVA methods, the LightGBM feature selection method can search for the optimal feature subset faster, and its corresponding model performance evaluation metrics are better. Finally, the BO algorithm is used to adjust the parameters of the LightGBM classifier to establish the best model. The results show that the IFS-LightGBM (BO) model is a very effective way to predict succinylation sites because of owing ACC of 0.7392, recall of 0.7219, MCC of 0.4771, precision of 0.7291, and *F*-measure of 0.7255.

## Figures and Tables

**Figure 1:** The overall framework of IFS-LightGBM (BO) for succinylation site prediction.

**Figure 2:** (a) Describes the IFS curve of the ACC value of each feature selection method, and (b) describes the IFS curve of the *F*-measure value of each feature selection method. According to the constructed dataset described in Materials and Methods, the IFS curve shows the trend of (a) ACC value and (b) *F*-measure value of the five feature selection methods as the number of input features increases. The five feature selection methods are LightGBM, ReliefF, LinearSVR, XGBoost, and ANOVA.

**Figure 3:** IFS curve describing the ACC value and *F*-measure value of each classifier. On the basis of the dataset constructed as described in Materials and Methods, the IFS curve shows the trend of the (a) ACC values and (b) *F*-measure values of the seven classifiers as the number of input features increases. The seven classification algorithms are LightGBM, Random Forest, ExtraTree, GBDT, kNN, XGBoost, and NB.

**Figure 4:** The maximum *F*-measure value distribution obtained by the different classifiers for 100 random tests is shown. The *x*-coordinate represents the maximum *F*-measure value, and the *y*-coordinate represents the number of corresponding intervals. The seven classifiers are (a) LightGBM, (b) Random Forest, (c) ExtraTree, (d) GBDT, (e) kNN, (f) XGBoost, and (g) NB.

**Figure 5:** Distributions of the top 351 features in the LightGBM feature list on four feature types. Figures (a), (b), and (c) show the distribution of the four types of features ranked in the top 100, top 101-200, and top 201-351 in the feature list, respectively.

**Table 1:** Distribution of 2501-dimensional features on four typical feature types.

Features	Feature description	Feature dims
CKSAAP	Short sequence motif information of polypeptide segments	2000
Disorder	Protein intrinsic disorder score	21
PseAAC	Physicochemical characteristics of amino acid factors	40
PSSM	Evolutionary information of amino acid residues	440
Total	—	2501

**Table 2:** Performance table for instances labeled with a class label A.

	True label A	True not A
Predicted label A	True positive (TP)	False positive (FP)
Predicted not A	False negative (FN)	True negative (TN)

**Table 3:** Predictive metrics of different feature extraction methods.

Features	Dimensional	ACC	Recall	MCC	Precision	*F*-measure
PseAAC	40	0.7061	0.6970	0.4113	0.6904	0.6937
Disorder	21	0.5709	0.5906	0.1434	0.5469	0.5679
CKSAAP	2000	0.6964	0.6849	0.3916	0.6810	0.6829
PSSM	440	0.6985	0.6576	0.3950	0.6947	0.6756
All	2501	0.7253	0.7053	0.4492	0.7153	0.7103
All (IFS)	2501	0.7360	0.7223	0.4708	0.7240	0.7232

**Table 4:** Predictive metrics of different feature selection methods.

Feature selection methods	Optimal subsets	ACC	Recall	MCC	Precision	*F*-measure
LightGBM	351	0.7360	0.7223	0.4708	0.7240	0.7232
ReliefF	2314	0.7319	0.7150	0.4626	0.7211	0.7181
LinearSVR	2107	0.7304	0.7114	0.4594	0.7204	0.7159
XGBoost	563	0.7351	0.7231	0.4692	0.7224	0.7228
ANOVA	1203	0.7316	0.7142	0.4620	0.7211	0.7176
*t*-SNE	3	0.5526	0.5112	0.1019	0.5328	0.5218
PCA	1517	0.6952	0.6617	0.3885	0.6880	0.6746

**Table 5:** Predictive metrics of respective feature subsets classified by each classifier.

Classifier	Optimal subsets	ACC	Recall	MCC	Precision	*F*-measure
LightGBM	351	0.7360	0.7223	0.4708	0.7240	0.7232
RF	37	0.7182	0.6795	0.4345	0.7158	0.6972
ET	33	0.6010	0.5934	0.2013	0.5804	0.5868
GBDT	94	0.7267	0.7223	0.4528	0.7102	0.7162
kNN	32	0.6596	0.7209	0.3258	0.6242	0.6691
XGBoost	427	0.7271	0.7114	0.4529	0.7154	0.7134
NB	805	0.6878	0.7724	0.3867	0.6444	0.7026

**Table 6:** The average and standard deviation of the maximum ACC of different classifiers.

Classifier	Max_ACC mean	Max_ACC std	Max of Max_ACC
LightGBM	0.7290	0.0027	0.7360
RF	0.7148	0.0023	0.7203
ET	0.5960	0.0049	0.6081
GBDT	0.7250	0.0021	0.7296
kNN	0.6614	0.0021	0.6661
XGBoost	0.7177	0.0032	0.7271
NB	0.6923	0.0008	0.6944

**Table 7:** The average and standard deviation of the maximum *F*-measure of different classifiers.

Classifier	Max_*F*-measure mean	Max_*F*-measure std	Max of Max_*F*-measure
LightGBM	0.7145	0.0029	0.7232
RF	0.6932	0.0027	0.6989
ET	0.5718	0.0060	0.5868
GBDT	0.7128	0.0022	0.7194
kNN	0.6677	0.0020	0.6730
XGBoost	0.7034	0.0035	0.7134
NB	0.7017	0.0009	0.7039

**Table 8:** Hyperparameter optimization results of IFS-LightGBM (BO).

Hyperparameters	Meanings	Search ranges	Optimal values
learning_rate	Learning rate	(0.01, 1.0)	0.0274
max_depth	Maximum depth of the tree	(1, 50)	20
max_bin	The max number of bins that feature values will be bucketed in	(10, 100)	10
reg_alpha	L1 regularization	(1*e*-9, 1.0)	0.9647
boosting_type	Training method	gbdt; goss; rf; dart	goss
num_leaves	Number of leaf nodes	(1, 50)	11
n_estimators	Number of iterations	(100, 600)	600

**Table 9:** Hyperparameter optimization results of LightGBM (GS).

Hyperparameters	Meanings	Search ranges	Optimal values
learning_rate	Learning rate	(0.01, 1.0)	0.1
max_depth	Maximum depth of the tree	(1, 50)	15
max_bin	The max number of bins that feature values will be bucketed in	(10, 100)	20
reg_alpha	L1 regularization	(1*e*-9, 1.0)	1*e*-5
boosting_type	Training method	gbdt; goss; rf; dart	gbdt
num_leaves	Number of leaf nodes	(4, 50)	36
n_estimators	Number of iterations	(100, 600)	450

**Table 10:** Performance comparison of IFS-LightGBM (BO), LightGBM, and LightGBM (GS).

Classifier	Optimal subsets	ACC	Recall	MCC	Precision	*F*-measure
IFS-LightGBM (BO)	351	0.7392	0.7219	0.4771	0.7291	0.7255
LightGBM	351	0.7360	0.7223	0.4708	0.7240	0.7232
LightGBM (GS)	351	0.7377	0.7190	0.4740	0.7282	0.7235

**Table 11:** The average and standard deviation of the maximum *F*-measure of IFS-LightGBM (BO), LightGBM, and LightGBM (GS).

Classifier	Max_*F*-measure mean	Max_*F*-measure std	Max of Max_*F*-measure
IFS-LightGBM (BO)	0.7229	0.0028	0.7292
LightGBM	0.7145	0.0029	0.7232
LightGBM (GS)	0.7194	0.0027	0.7259

## Data Availability

The data used to support the findings of this study are from previously reported studies and public database, which have been cited.
